# Determinants of access to improved sanitation facilities in rural districts of southern Ghana: evidence from Dodowa Health and Demographic Surveillance Site

**DOI:** 10.1186/s13104-018-3572-6

**Published:** 2018-07-13

**Authors:** David Etsey Akpakli, Alfred Kwesi Manyeh, Jonas Kofi Akpakli, Vida Kukula, Margaret Gyapong

**Affiliations:** 1 Ghana Health Service/Dodowa Health Research Centre, Dodowa, Ghana; 2 University of Health and Allied Sciences, Ho, Ghana; 3 Ubora Institute, Accra, Ghana; 4 School of Public Health, University of the Witwatersrand, Johannesburg, South Africa

**Keywords:** Household head, Improved sanitation, Rural, Ghana

## Abstract

**Objective:**

Access to improved sanitation facilities is critical to the health and well-being of individuals and communities. However, globally, over 2.5 billion people live without access to safe sanitation facilities and more than 40% of the world population, do not use a toilet, but defecate in the open or in unsanitary places. In Ghana, only 14% of the population have access to improved sanitation facilities with great disparities between rural (8%) and urban (19%) dwellers. This paper sought to examine the determinants of access to improved sanitation facilities by households among rural dwellers in two districts in southern Ghana.

**Results:**

This study, which involved 16,353 household heads from the Dodowa Health and Demographic Surveillance System, found that sanitation facilities used by households were significantly influenced by age, gender, level of education, occupation, marital and socioeconomic status of household heads. It further revealed that a large proportion (85.94%) of the study participants did not have access to improved sanitation facilities. The study therefore recommends that the national sanitation laws must strictly be enforced to ensure each household in Ghana has decent and hygienic toilet facility.

## Introduction

Basic sanitation is considered the lowest-cost technology ensuring hygienic excreta disposal and a clean and healthful living environment both at home and in the neighborhood of users [1]. It involves the use of improved sanitation facilities such as public sewer connection; septic system connection; pour-flush latrine; simple pit latrine; ventilated improved pit latrine and private facilities (sanitation facilities used exclusively by a household) [1]. According to WHO, only private facilities are considered to be improved [2]. The goal of improved sanitation is to hygienically separate human excreta from human contact and therefore reduce exposure to fecal contamination [3, 4]. By WHO standards, even an improved facility that is shared by more than one household is considered unimproved [4, 5].

Globally, over 2.5 billion people are living without access to safe sanitation facilities which leads to about 200 million tonnes of untreated human excreta annually [6, 7]. About 2.6 billion people, more than 40% of the world population, do not use toilet facilities, but defecate in the open or in unsanitary places [2]. Access to improved sanitation facilities is a huge challenge in Africa. In Nigeria, over 130 million people, two-thirds of the population, do not have access to adequate sanitation facilities [8] whilst in South Africa about 18 million people also face the same challenge [9]. More than half the population of Ghana (59%), the highest in the world, depend on shared sanitation facilities including public toilets [10] and about 19% of Ghanaians practise open defecation while 8% depend on various forms of unimproved sanitation facilities options such as bucket latrines [8].

This paper sought to explore the determinants of access to improved sanitation facilities by households among rural dwellers in the Dodowa Health and Demographic Surveillance area.

## Main text

### Methods

#### Study site and population

Data for this study was extracted from Dodowa Health and Demographic Surveillance System (DHDSS) which is located in the south-eastern part of Ghana. The operation of the DHDSS can be found elsewhere [10].

The study population comprised household heads (HHs) that were resident in the DHDSS from January 1, 2013 to December 31, 2013.

#### Outcome and exposure variables

The outcome variable for this study was type of sanitation facility which is binary and was recorded as 1 “improved” and 0 “unimproved”. The unimproved sanitation facilities included open defecation (use of bush or beach), shared pit latrine, own pit latrine and shared ventilated improve pit latrine while the improved sanitation facilities included the use of own ventilated improved pit latrine and flush toilet.

From the available data, seven [7] exposure variables were selected: age, sex, level of education, occupation, marital status, household size and socioeconomic status (wealth index) of the HHs. These exposure variables were selected because from available literature, they have the potential to influence the type of sanitation facilities used by households. The wealth index is a proxy measure of a household’s long term standard of living derived through principal component analysis [11].

#### Statistical analysis

The extracted data were cleaned to identify all missing values and to check for internal consistency of the responses. Any irregularities in the data were corrected by using the hard copies of the completed questionnaires. Variables were recoded where necessary. The relationship between each exposure variable and outcome variable were explored at the univariate and multivariate level using logistic regression. All analyses were conducted in STATA version 11. The results were presented in the form of tables and summary statistics in odds ratios (OR), with 95% confidence intervals (CI) and P-values.

### Results

#### Background characteristics

Table 1 provides the descriptive information on the socio-demographic characteristics of 16,353 HHs who were included in the study. The median age of the HHs was 48 years (IQR = 23). The majority (73.71%) of the HHs were of the Ga-Dangme ethnic group and 60.46% were male. A little more than half of HHs (52.72%) had junior or senior high school and above level of education while about one-thirds (33.89%) had no formal education. Of the HHs that were studied, 37.34% were married whereas 7.94% were divorced/separated. About two-fifths (40.84%) of the HHs were farmers, while 6.37% were unemployed. The study found that about one-quarter (26.33%) had a household size of six and more. The majority of the HHs (85.94%) studied used unimproved sanitation facilities.

**Table 1:** Socio-demographic characteristics of the study participants

	Frequency	Percentage (%)
Age group		
< 30	1068	6.53
30–34	1644	10.05
35–39	2046	12.51
40–44	2058	12.58
45–49	1861	11.38
50–54	1806	11.04
55–59	1446	8.84
60–64	1259	7.70
65–69	889	5.44
70+	2276	13.92
Median = 48 (IQR = 23)		
Sex		
Female	6466	39.54
Male	9887	60.46
Ethnicity		
Ga-Dangme	12,054	73.71
Akan	1007	6.16
Ewe	2511	15.35
Northern	675	4.13
Others	106	0.65
Marital status		
Single	1772	10.84
Divorced/separated	1298	7.94
Married	6107	37.34
Cohabiting	5307	32.45
Widowed	1869	11.43
Education		
No education	5542	33.89
Primary	2189	13.39
Junior high/middle school	5886	35.99
Senior high school and above	2736	16.73
Occupation		
Unemployed	1041	6.37
Farmer	6678	40.84
Artisan	2917	17.84
Trader	2987	18.27
Civil servant	1007	6.16
Fisherman	797	4.87
Others	926	5.66
Household size		
Less than six	12,047	73.67
Six and above	4306	26.33
Sanitation (toilet) type		
Unimproved	14,053	85.94
Improved	2300	14.06

#### Bivariate analysis

From Table 2, 90.98 and 82.63% of the households headed by females and males used unimproved sanitation facilities, respectively. A total of 34.72% of HHs with senior high school and above level of education used improved sanitation facilities while those with junior/middle school education constituting 14.51% of the study population used improved sanitation facilities. Only 5.88% households who had no formal education used improved sanitation facilities whilst those with primary level of education constituted 7.77%.

**Table 2:** Bivariate analysis of determinants of improved and unimproved sanitation facilities used by households

Characteristics of household head	Unimproved n (%)	Improved n (%)	*P* value
Age group			
< 30	958 (89.70)	110 (10.30)	< 0.001
30–34	1473 (89.60)	171 (10.40)	
35–39	1795 (87.73)	251 (12.27)	
40–44	1779 (86.44)	279 (13.56)	
45–49	1562 (83.93)	299 (16.07)	
50–54	1514 (83.83)	292 (16.17)	
55–59	1172 (81.05)	274 (18.95)	
60–64	1057 (83.96)	202 (16.04)	
65–69	725 (81.55)	164 (18.45)	
70+	2018 (88.66)	258 (11.34)	
Sex			
Female	5883 (90.98)	583 (9.02)	< 0.001
Male	8170 (82.63)	1717 (17.37)	
Ethnicity			
Ga-Dangme	10,741 (89.11)	1313 (10.89)	< 0.001
Akan	643 (63.85)	364 (36.15)	
Ewe	2029 (80.80)	482 (19.20)	
Northern	5,58 (82.80)	117 (17.33)	
Others	82 (77.36)	24 (22.64)	
Marital status			
Single	1524 (86.00)	248 (14.00)	< 0.001
Divorced/separated	1151 (88.67)	147 (11.33)	
Married	4963 (81.27)	1144 (18.73)	
Cohabiting	4726 (89.05)	581 (10.95)	
Widowed	1689 (90.37)	581 (9.63)	
Level of education			
No education	5216 (94.12)	326 (5.88)	< 0.001
Primary	2019 (92.23)	170 (7.77)	
Junior high/middle school	5032 (85.49)	854 (14.51)	
Senior high school and above	1786 (65.28)	950 (34.72)	
Occupation			
Unemployment	925 (88.86)	116 (11.14)	< 0.001
Farmer	6022 (90.18)	656 (9.82)	
Artisan	2449 (83.96)	468 (16.04)	
Trader	2697 (90.29)	290 (9.71)	
Civil servant	612 (60.77)	395 (39.23)	
Fisherman	662 (83.06)	135 (16.94)	
Others	686 (74.08)	240 (25.92)	
Household size			
Less than six	10,377 (86.14)	1670 (13.86)	0.213
More than five	3676 (85.37)	630 (14.63)	
Socioeconomic status			
Poorest	705 (99.44)	4 (0.56)	< 0.001
Poorer	2017 (97.25)	57 (2.75)	
Poor	3325 (94.11)	208 (5.89)	
Less poor	4334 (92.94)	329 (7.06)	
Least poor	3672 (68.33)	1702 (31.67)	

Ninety-nine percent (99.44%) of the households in the poorest socioeconomic quintile had unimproved sanitation facilities compared to 68.33% of the HHs in the least poor socioeconomic quintile. Statistically, there was an association (P < 0.05) between the variables studied and type of sanitation facility being used except for household size.

#### Univariate and Multivariate Analysis

From Table 3, male HHs were more than twice likely to use improved sanitation facilities compared to the female HHs and this was statistically significant. After adjusting for age group, marital status, education, occupation and socioeconomic status, sex of HHs was still associated with type of sanitation facility such that male HHs were 1.23 times more likely to use improved sanitation facilities compared to the female headed households.

**Table 3:** Unadjusted and adjusted odd ratios of determinants of improved and unimproved sanitation facilities used by households

Characteristics	Unadjusted			Adjusted		
	OR	95% CI	P-value	OR	95% CI	P-value
Age group						
< 30	1.00			1.00		
30–34	1.01	0.79–1.30	0.932	0.99	0.75–1.30	0.938
35–39	1.22	0.96–1.54	0.104	1.21	0.93–1.58	0.157
40–44	1.37	1.08–1.73	0.009	1.60	1.22–2.09	0.001
45–49	1.67	1.32–2.10	< 0.001	2.01	1.53–2.62	< 0.001
50–54	1.68	1.33–2.12	< 0.001	2.23	1.70–2.93	< 0.001
55–59	2.04	1.61–2.58	< 0.001	2.73	2.06–3.60	< 0.001
60–64	1.66	1.30–2.13	< 0.001	2.71	2.02–3.62	< 0.001
65–69	1.97	1.52–2.56	< 0.001	3.32	2.44–4.51	< 0.001
70+	1.11	0.88–1.41	0.372	3.02	2.27–4.03	< 0.001
Sex						
Female	1.00			1.00		
Male	2.12	1.92–2.34	< 0.001	1.23	1.05–1.38	0.008
Education						
No education	1.00			1.00		
Primary	1.35	1.11–1.63	0.002	1.28	1.04–1.58	0.019
Junior high/middle school	2.72	2.38–3.10	< 0.001	1.73	1.48–2.03	< 0.001
Senior high school and above	8.51	7.42–9.76	< 0.001	3.28	2.74–3.91	< 0.001
Marital status						
Single	1.00			1.00		
Divorced/separated	0.78	0.63–0.98	0.029	0.97	0.75–1.25	0.826
Married	1.42	1.22–1.64	< 0.001	1.06	1.88–1.27	0.557
Cohabiting	0.76	0.64–0.89	0.001	0.85	0.71–1.02	0.080
Widowed	0.65	0.53–0.80	< 0.001	0.81	0.63–1.03	0.090
Household size						
Less than six	1.00					
Six and above	1.06	0.96–1.18	0.213			
Occupation						
Unemployed	1.00			1.00		
Farmer	0.87	0.70–1.07	0.187	0.93	0.73–1.17	0.526
Artisan	1.52	1.23–1.89	< 0.001	1.05	0.82–1.35	0.691
Trader	0.86	0.68–1.08	0.186	1.00	0.77–1.28	0.983
Civil servant	5.15	4.09–6.48	< 0.001	1.57	1.21–2.05	0.001
Fisherman	1.63	1.24–2.12	< 0.001	1.31	0.97–1.77	0.084
Others	2.79	2.19–3.55	< 0.001	1.62	1.23–1.24	0.001
Socioeconomic status						
Poorest	1.00			1.00		
Poorer	4.98	1.80–13.77	0.002	4.91	1.77–13.61	0.002
Poor	11.03	4.09–29.75	< 0.001	10.66	3.94–28.81	< 0.001
Less poor	13.38	4.98–35.98	< 0.001	11.40	4.23–30.74	< 0.001
Least poor	81.69	30.52–218.64	< 0.001	52.44	19.52–140.89	< 0.001

Household heads aged 40–44, 45–49, 50–54, 55–59, 60–64, 65–59 years were at least 36% more likely to use improved sanitation facilities compared to those aged less than 30 years. This was still significant after controlling for sex, marital status, education, occupation and socioeconomic status.

While HHs with primary level of education were 1.35 times more likely to use improved sanitation facilities compared to those with no formal education in the unadjusted model, those with junior high/middle and senior high school and above level of education were 2.72 and 8.51 times more likely to use improved sanitation facilities, respectively compared to those with no formal education. This was statistically significant.

Also, while HHs who were married were 1.42 times more likely to use improved sanitation facilities, those who were divorced/separated, cohabiting and widowed were 22, 24 and 35% less likely to use improved sanitation facilities, respectively compared to those who were single. This was also statistically significant in the unadjusted model. After adjusting, none of them was statistically significant.

Households with more than five members were 1.06 times more likely to use improved sanitation facilities compared to those with less than six members in the unadjusted model and this was statistically not significant.

Civil Servants were 5.15 times more likely to use improved sanitation facilities compared to HHs who were unemployed. This association was significant in both the unadjusted and adjusted models. Artisans and fishermen were 1.52 and 1.63 times more likely to use improved sanitation facilities, respectively compared to HHs who were unemployed. Farmers and petty traders were 13 and 14% less likely to use improved sanitation facilities, respectively compared to HHs who were unemployed.

Household heads with poorer, poor, less poor and least poor socioeconomic status were 4.98, 11.03, 13.38 and 81.69 times more likely to use improved sanitation facilities, respectively compared to HHs from the poorest households. This was still statistically significant after adjusting for other explanatory variables.

### Discussion

#### Household demographics

The age distribution of most HHs (57.57%) was found to be between 30 and 54 years. This indicates that the HHs within the study area fell within the economically active group [12]. A large proportion (60.46%) of HHs were males which reinforces the belief that men generally are considered heads of the family units. Studies by Ridgeway and Smith-Lovin [13], Lewis [14] and Salomone [15] confirmed this assertion [16].

#### Socio-demographic determinants

The findings revealed that only 14.06% of the HHs studied used improved sanitation facilities. This figure agrees with the national figure of 14.00% [17]. Unimproved sanitation facilities have economic, social, cultural, sex, health, environmental and income effects and to a large extent impede the full realization of human development of the affected persons [16]. Diseases related to poor sanitation and lack of hygiene are some of the most common causes of illness and death among the poor of developing countries [18].

Results of our study showed that HHs aged between 40 and 69 years were at least 36% more likely to use improved sanitation facilities compared to those aged less than 30 years. This could mean that majority of the said category of the study population fall within the economically active group and could afford improved sanitation facilities. A study by Angko revealed similar finding [16].

For sex distribution, the study result showed that male HHs were more than twice likely to use improved sanitation facilities compared to the female HHs. In most societies, women have the primary responsibility for management of household water, sanitation and health. They spend much time on household chores which reinforces time-poverty, disempowers them and lowers their income [19]. In fact this affects the socioeconomic and health conditions of the women in many ways [20].

Further, the findings indicated that the higher the level of education of HHs, the more likely they were to use improved sanitation facilities. This is consistent with a study carried out by Koskei which revealed that educational level of HH has close relationship with access and use of sanitation facilities [21]. From the findings of this study, about one-thirds of the study population had no formal education. This could explain why majority of them used unimproved sanitation facilities. Nonetheless, these findings contradict the Ghana multiple indicator cluster survey which shows no significant association [22].

For marital status, a study by Koskei revealed similar findings as our study where, most of the married respondents studied, used improved sanitation facilities and only 14% of those who were separated used improved sanitation facilities. None of the study participants who were single and widowed used improved facilities [21].

#### Socio-economic determinants

Civil Servants were more likely to use improved sanitation facilities compared to HHs who were unemployed. Interestingly, our study found that artisans and fishermen were more likely to use improved sanitation facilities whilst farmers and petty traders were less likely to use improved sanitation facilities compared to HHs who were unemployed. It was also found that access to improved sanitation facilities was mostly determined by the wealth of the households such that the poorer the socioeconomic status of HHs, the less likely it was they would use improved sanitation facilities. According to Boadi and Kuitunen [23], household wealth played a vital role in the acquisition and utilization of improved toilet facilities because of the correlation between household wealth and access to improved well-being [24]. Wealthy households were in a better position to provide improved toilet facilities for their members whilst poor households who were fortunate to have toilet facilities usually shared with other households [24].

This study concludes that age, gender, level of education, occupation, marital and socioeconomic status of HHs are significant determinants of the type of sanitation facilities used and that a large proportion of residents within the study area resort to the use of unimproved sanitation facilities. To meet the Sustainable Development Goal of achieving universal access to improved sanitation facilities and to eliminate open defecation by 2030, our study recommends that city authorities must strictly enforce the national sanitation laws which state that all households in Ghana must have decent and hygienic toilet facilities in their homes/compounds.

## Limitations

Although this study used a large sample size, its findings are unlikely to be generalized since the HDSS covers only two districts out of the 216 districts in Ghana. Also, other important variables such as culture, traditions, social norms, etc. which could equally have influence on the use of sanitation facility type were not available in the HDSS data.

## Abbreviations

CLTS: Community-Led Total Sanitation
DWD: Dangme West District
DHDSS: Dodowa Health and Demographic Surveillance System
DHRC: Dodowa Health Research Centre
GDHS: Ghana Demographic Health Survey
GHS: Ghana Health Service
GSS: Ghana Statistical Service
INDEPTH: International Network for the Demographic Evaluation of Populations and Their Health
MDG: Millennium Development Goal
MLGRD: Ministry of Local Government and Rural Development
MICS: Multiple Indicator Cluster Survey
UNICEF: United Nations Children’s Fund
WHO: World Health Organization
